The article "Early Postoperative Pain Control and Inflammation for Total Knee Arthroplasty: A Retrospective Comparison of Continuous Adductor Canal Block versus Single-Shot Adductor Canal Block Combined with Patient-Controlled Intravenous Analgesia" was retracted in 2024. Reasons: signs of a paper mill; suspected computer-generated content; unreliable results or conclusions; concerns about the data.

# Early Postoperative Pain Control and Inflammation for Total Knee Arthroplasty: A Retrospective Comparison of Continuous Adductor Canal Block versus Single-Shot Adductor Canal Block Combined with Patient-Controlled Intravenous Analgesia

**DOI:** 10.1155/2022/1351480

**Published:** 2022-05-11

**Authors:** Xiaojuan Yang, Jun Dong, Wei Xiong, Fusen Huang

**Affiliations:** The Department of Anesthesiology, The First Affiliated Hospital of Chongqing Medical University, Chongqing, China

## Abstract

**Objective:**

The aim of this study was to compare pain control and inflammation among patients who received a continuous adductor canal block (CACB) versus single-shot adductor canal block (SACB) combined with patient-controlled intravenous analgesia (PCIA) for total knee arthroplasty (TKA) analgesia in the first two days after surgery.

**Design:**

Matched cohort retrospective study. *Setting*. University hospital. *Patients*. One hundred fifty-six patient charts were included in this study: 78 patients with CACB in Group A and 78 patients with SACB combined with PCIA in Group B. Patients were matched according to age, body mass index, and American Society of Anesthesiologists class. *Measurements*. The primary outcome of the study was Visual Analogue Scale (VAS) pain scores before operation (Pre) and at postoperative 6 (POH6), 12 (POH12), 24 (POH24), 30 (POH30), 36 (POH36), and 48 hours (POH48). Secondary outcomes included patient-controlled bolus, time of first postoperative ambulation, range of knee flexion and extension, inflammation cytokines on Pre and POH48, percentage of remedial analgesics treatment, incidence of adverse events and complications, hospital stay and cost, and Numerical Rating Scale (NRS) satisfaction scores at discharge. *Main Results*. Mean VAS scores at rest and with motion were lower in Group B than in Group A on all postoperative hours. At POH30, compared with Group A (1.1 ± 0.6), mean VAS scores at rest in Group B (0.9 ± 0.4) were lower (*P*=0.048), and compared with Group A (2.6 ± 0.7), mean VAS scores with motion in Group B (2.2 ± 0.8) were lower (*P*=0.001). The number of patient-controlled bolus was 4.3 ± 1.6 (95% CI 3.9–4.6) in Group A and 3.1 ± 1.3 (95% CI 2.8–3.4) in Group B, respectively (*P* < 0.001). Patients in Group B displayed better functional recovery and inflammation results at POH48 than Group A with respect to range of knee flexion and extension (117.8 ± 10.9° vs. 125.2 ± 9.4°, *P* < 0.001) and inflammation cytokines, including erythrocyte sedimentation rate (ESR), C-reactive protein (CRP), and interleukin-6 (IL-6) ((43.8 ± 16.1) vs. (36.8 ± 13.2), *P*=0.003; (34.9 ± 9.4 mg/L) vs. (29.6 ± 10.6 mg/L), *P*=0.001; (21.3 ± 8.7 pg/ml) vs. (14.0 ± 7.0 pg/ml), *P* < 0.001)).

**Conclusion:**

SACB combined with PCIA in the first two days of patients undergoing TKA has better analgesic and beneficial effects on functional recovery and inflammation.

## 1. Introduction

Total knee arthroplasty (TKA) is currently an advanced and effective method for the treatment of knee osteoarthritis. In the early stage after TKA, patients suffered from moderate to severe pain [1, 2] and obvious inflammation, which was manifested by the obvious increase in inflammatory cytokines such as interleukin-6 (IL-6), C-reactive protein (CRP), and erythrocyte sedimentation rate (ESR) [3, 4]. However, persistent postoperative pain and inflammation impair patients from achieving the desired knee joint function recovery after TKA [5].

Many modalities, such as adjuvant analgesic agents, patient-controlled intravenous analgesia (PCIA), epidural analgesia [6], periarticular infiltration, and peripheral nerve block [7–10], are used for pain relief after TKA. There is a growing consensus now that adductor canal block (ACB) was an effective method for analgesia management after TKA [9–13], which could reduce opioid dosage [12] and was conducive to knee joint function rehabilitation [10, 13]. Canbek et al. had reported that CACB provided a better analgesia compared to a single-shot adductor canal block (SACB) after TKA [14–16]. The nonsteroidal anti‐inflammatory drugs (NSAIDs) not only relieved pain but also inhibited inflammation. Zhuang et al. had found that IL-6, ESR, and CRP levels were reduced in the parecoxib/celecoxib group after TKA [17].

Data related to orthopedic patients have been recorded since enhanced rehabilitation after surgery (ERAS) was performed in our hospital in April 2016. From February 2019 to June 2020, the ERAS team in our orthopedics department implemented CACB to control pain for TKA patients. Nevertheless, perioperative analgesia for TKA patients should not only relieve pain but also pay attention to the occurrence of inflammation. Due to the analgesic and anti-inflammatory effects of NSIADs in PCIA, our team adjusted the analgesic regimen to SACB combined with PCIA from July 2020 to May 2021. However, we still have no idea about whether there was a difference in the postoperative analgesia and inflammation between CACB and SACB combined with PCIA after TKA. The objective of this work was to compare two different analgesic protocols applied to patients who underwent unilateral primary total knee arthroplasty and analyze the quality of pain control, inflammation, hospital stay, and cost, in order to enhance recovery after surgery.

## 2. Materials and Methods

Institutional review board approval was obtained for this research. As this trial was retrospective in nature, neither written informed consent nor clinical trial registration were required.

A total of 300 patient charts were screened for review from February 2019 to May 2021, and we retrospectively analyzed the anesthesia record list, hospital chart, and the iPainfree system, which was the pain management information system used for recording the patient-controlled analgesia (PCA) follow-up data. Patients who met the following criteria were excluded: (1) long-term abuse of opioids; (2) preexisting neuropathy in the ipsilateral lower extremity; (3) incomplete documentation for any of the primary or secondary outcome variables; (4) received bilateral TKA and/or other procedures; (5) transferred to the rehabilitation department to continue rehabilitation treatment without discharge; (6) accompanied by coagulation abnormalities or severe central nervous system diseases. Qualifying patients were matched according to age (18–90 years old), body mass index (BMI) (18–35 kg/m^2^), and American Society of Anesthesiologists (ASA) class (grade II-III). After this screening process, we recruited 156 patients who underwent a primary, selective, and unilateral TKA for knee osteoarthritis with general anesthesia by five orthopedic surgeons and two anesthesiologists in this study. 78 patients had CACB in Group A, and 78 patients had SACB combined with PCIA in Group B.

### 2.1. Outcome Measures

The following demographic and perioperative data were collected: gender, age, height, weight, BMI, ASA class, medical history, operation procedure, operation time, anesthesia method and content, intraoperative medication, anesthesia time, postoperative analgesia protocol, time of extubation, and length of stay in the postanesthesia care unit (PACU).

The primary outcomes of the study were Visual Analogue Scale (VAS) pain scores before operation (Pre) and at postoperative 6 hours (POH6), 12 hours (POH12), 24 hours (POH24), 30 hours (POH30), 36 hours (POH36), and 48 hours (POH48) at rest and motion. Nerve block catheters and PCIA were discontinued at POH48.

Secondary outcomes were time of first postoperative ambulation; range of knee flexion and extension; inflammation cytokines at Pre and POH48, including erythrocyte sedimentation rate (ESR), C-reactive protein (CRP), and interleukin-6 (IL-6); incidence of adverse events (including patient-controlled bolus, dizziness, nausea and vomiting, and remedial analgesics treatment) and complications (including pulmonary infection, cardiovascular events, deep vein thrombosis, incisional infection, and unplanned second surgery); postoperative hospital stay, total hospital stay, total hospital cost, and patient self-reported satisfaction score at discharge. Numerical Rating Scale (NRS) was scored with range 0–10, 0 = not at all satisfied and 10 = very satisfied.

### 2.2. Intraoperative Course

Patients took celecoxib 200 mg orally daily for advanced analgesia and, if there were no contraindications, had low-molecular-weight heparin anticoagulation after admission. Before surgery, patients abstained from food for 8 h and drinking for 2 h but drank the nutrition solution prepared by the nutrition department on the day of surgery.

Patients were routinely monitored for electrocardiogram, blood pressure, pulse oxygen saturation, respiratory rate, and temperature during the perioperative period. After general anesthesia induction, endotracheal intubation and mechanical ventilation were performed. Anesthesia was maintained with sevoflurane inhalation and intravenous infusion of propofol and remifentanil, and vecuronium was added intermittently as needed. Intravenous injection of dexamethasone (10 mg) and tropisetron (2 mg) was performed to prevent postoperative nausea and vomiting. Five different surgeons performed the procedures, and then, two different senior anesthetists performed adductor canal block on all patients immediately with the technique described by Jenstrup et al. [18]. After that, patients were transferred to PACU, the tracheal tube was removed when they reached the extubation indications, and then they were transferred to the ward.

Postoperative management measures included using parecoxib 40 mg daily for analgesia. Omeprazole for acid inhibition and gastric protection was used without contraindications. Low-molecular-weight heparin was used for preventing deep vein thrombosis. Cefuroxime was used for preventing infection and monitoring inflammation cytokines. Patients were encouraged to gradually resume their diet and lower limb activities 2 hours after surgery. Rehabilitation physicians guided rehabilitation training at POH6 and encouraged patients to get out of bed as soon as possible.

### 2.3. Postoperative Analgesia Course

#### 2.3.1. Group A

At the end of the operation, an adductor canal block was performed via guidance of ultrasound, injecting 20 ml 0.2% ropivacaine, and inserting a catheter, which was then properly fixed and connected to the electronic patient-controlled analgesic pump. Analgesic pump drugs in the CACB group were prepared with 300 ml of 0.17% ropivacaine. Analgesic pump parameters included load dose 5 ml; basal infusion rate 5 ml/h; patient-controlled bolus dose 5 ml; and security lock duration 45 minutes.

#### 2.3.2. Group B

Single-shot adductor canal block was performed under ultrasound guidance after surgery, injected with 20 ml 0.2% ropivacaine without catheterization, and then intravenous infusion of the PCIA was started. Analgesic pump drugs in PCIA were prepared with tramadol 800 mg combined with flurbiprofen axetil 100 mg and saline mixed into 80 ml. Analgesic pump parameters included load dose 5 ml; basal infusion rate 1 ml/h; patient-controlled bolus dose 2 ml; security lock duration 15 minutes.

Based on a load dose, the PCA pump started to work continuously at the end of the operation. The department of anesthesiology had special personnel for following up the patients who use PCA at 6 h, 12 h, 24 h, 30 h, 36 h, and 48 h after surgery. They completed the follow-up records through the iPainfree pain management information system. They collected and recorded the hemodynamic parameters, patient self-reported pain scores (Visual Analogue Scale, VAS), and the adverse events including time of patient-controlled bolus, dosage of PCA, remedial analgesics treatment, dizziness, nausea and vomiting, sedation score, pruritus, urinary retention, sensory disorder, dyskinesia, and local puncture anomaly. The specific method of VAS score is as follows: a 10 cm line segment was drawn on a paper. The left end of the line segment is 0 points, indicating no pain, and the right end is 10 points, indicating severe pain (the pain degree increases gradually from left to right). Patients in the calm state was marked according to the self-marking line segment, indicating the degree of pain. If VAS scores ≥4, patients in both groups were treated with remedial analgesia: paracetamol and tramadol and/or celecoxib and/or gabapentin.

### 2.4. Statistics

Statistical analysis was conducted using SPSS 26.0 (International Business Machines Corporation, USA) software. Conformity of the data to normal distribution was tested with the Kolmogorov–Smirnov test. Data are shown as mean ± standard deviation, or number (percentage). To determine statistical significance, the ANOVA test was used for testing VAS pain score, ESR, CRP, IL-6, patient-controlled bolus, the range of knee flexion and extension, postoperative hospital stay, and NRS satisfaction score. Pearson's chi square test was used for gender, ASA class, surgery side, and the incidence of adverse events and complications. *P* < 0.05 was considered as statistically significant.

## 3. Results

Between the CACB and SACB combined with the PCIA group, there was no significant difference in the demographic and perioperative data (Table 1; *P* > 0.05). As expected with our matching process, the percentage of the surgeons who performed surgery and the anesthetists who performed adductor canal block were no different. No neuropathic complications occurred in either group.

### 3.1. Pain Control

As shown in Figures 1 and 2, mean VAS scores at rest (1.1 ± 0.7 Group A vs. 1.0 ± 0.5 Group B, *P*=0.288) and with motion (2.8 ± 0.8 Group A vs. 2.6 ± 0.8 Group B, *P*=0.273) before operation were comparable. However, compared with Group A, the mean VAS scores at rest and with motion were lower in Group B at all postoperative hours. Compared with Group A, the mean VAS scores at rest (1.1 ± 0.6 vs. 0.9 ± 0.4, *P*=0.048) and with motion (2.6 ± 0.7 vs. 2.2 ± 0.8, *P*=0.001) in Group B were lower at POH30. The mean VAS scores at rest and with motion at POH6 and POH12 were lower than those before operation in both the groups (*P* < 0.012). The mean VAS scores at rest and with motion at POH12, POH24, POH30, POH36, and POH48 were higher than those at POH6 in both the groups (*P* < 0.015). The mean VAS scores at rest and with motion at POH24 and POH30 were higher than those at POH12 in both the groups (*P* < 0.04). The mean VAS scores with motion at POH36 were lower than those at POH30 in both the groups (*P* < 0.013).

The number of patient-controlled boluses was 4.3 ± 1.6 (95% CI 3.9–4.6) in Group A vs. 3.1 ± 1.3 (95% CI 2.8–3.4) in Group B, respectively (*P* < 0.01). There was no statistical difference between 9 patients (11.5%) in Group A and 5 patients (6.4%) in Group B using remedial analgesia (*P*=0.402).

### 3.2. Functional Recovery

As shown in Figure 3, the range of knee flexion and extension before operation (99.9 ± 12.4° in Group A vs. 101.8 ± 10.9° in Group B, *P*=0.323) was comparable. Compared with Group A, the range of knee flexion and extension at POH48 in Group B was higher, and the difference was statistically significant (117.8 ± 10.9° vs. 125.2 ± 9.4°, *P* < 0.001). Time of postoperative first ambulation was not statistically different (20.8 ± 4.1 h in Group A vs. 20.3 ± 3.9 h in Group B, *P*=0.448).

### 3.3. Inflammation Cytokines

As shown in Figures 4–6, mean ESR, CRP, and IL-6 were lower before operation as compared to POH48 (*P* < 0.001). Compared with Group A, mean ESR, CRP, and IL-6 in Group B at POH48 were lower and the difference were statistically significant ((43.8 ± 16.1) vs. (36.8 ± 13.2), *P*=0.003; (34.9 ± 9.4 mg/L) vs. (29.6 ± 10.6 mg/L), *P*=0.001; (21.3 ± 8.7 pg/ml) vs. (14.0 ± 7.0 pg/ml), *P* < 0.001)).

### 3.4. Economic Benefit

As shown in Tables 2 and 3, there was no significant difference in total hospital stay, incidence of dizziness, nausea and vomiting, pulmonary infection, and deep vein thrombosis between the two groups. Postoperative hospital stay was different between the two groups (*P* < 0.001), estimated about 1.1 day less following the use of SACB combined with PCIA. The total hospital cost was different between the two groups (*P*=0.001), estimated about 4032 RMB less following the use of SACB combined with PCIA. Compared with Group A, NRS satisfaction scores in Group B were higher at discharge and the difference was statistically significant (9.5 ± 0.3 vs. 9.7 ± 0.2, *P* < 0.001). Complications of cardiovascular events, incisional infection, and unplanned second surgery did not occur in either group.

## 4. Discussion

In this study, we found that the combination of SACB and PCIA was more effective than CACB alone in the management of early postoperative pain after TKA. VAS scores at rest in almost all postoperative hours and VAS scores with motion at all postoperative hours in both the groups were significantly lower than preoperation VAS scores, which indicated that both CACB and SACB combined with PCIA could effectively control the postoperative pain after TKA. Remarkably, the CACB group seemed to be the least beneficial modality of the two, which had the higher rest and motion VAS scores in all postoperative hours and needed more supplemental patient-controlled bolus and remedial analgesics treatment. There was a strong trend toward superiority of the SACB combined with PCIA group over CACB at POH30. The time of first postoperative ambulation was 15–30 hours after surgery in 90% patients in both the groups, and the VAS scores were significantly higher at POH24 and POH30 compared with POH6. It was not hard to see that the trend of VAS scores was likely related to postoperative rehabilitation training and movement [19, 20] in both groups. Like any continuous blockade technique, we ascribed CACB fared so poorly in this trial to secondary block failure [21, 22] or catheter displacement [23].

Severe pain was present after TKA [1, 2, 19] and lasted for 2-3 days after surgery [24]. A multimodal pain management protocol [9, 12, 13, 25, 26] after TKA has been shown to decrease narcotic usage [21], improve pain score/satisfaction, and facilitate joint early function rehabilitation [6, 24] over traditional patient-controlled intravenous analgesia (PCIA) alone [12, 27]. Canbek et al. showed that pain control following TKA was found to be superior in the patients given CACB compared with SACB, with better ambulation and functional recovery, and that SACB alone was not recommended to be used as an analgesia method [14]. According to the previous studies, the ERAS team in our orthopedics department implemented CACB or SACB combined with PCIA for TKA postoperative analgesia. To our knowledge, this was the first study to investigate pain control in patients received SACB when used in combination with PCIA in the first two days after TKA. All the adductor canal blocks in this study were performed by two experienced anesthetists with ultrasound visualization of both the catheter tip and local anesthetic spread during the initial bolus. In addition, multimodal analgesic treatment for all patients in our study started from admission, and systematic pain management was carried out throughout the perioperative period.

As we all know, the concentration and dose of local anesthetics have a great influence on the effect and duration of nerve block and that increasing the concentration and dose of local anesthetics carries the risk of causing systemic toxicity. The concentration of ropivacaine used for adductor canal block has been reported to vary widely from 0.1% to 0.75% [20, 28, 29], and the dosage of ropivacaine also varies widely from 5 ml to 40 ml [10, 15, 30, 31]. Wang et al. had found that EV50 of 0.5% ropivacaine for ACB was 10.79 ml (95% CI 10.10–11.52 ml) [32]. Christiansen et al. had found that no effect of increasing the volume of ropivacaine 0.2% from 5 to 30 ml on sensory sciatic nerve block duration [33]. It was not hard to see that the use of 20 ml 0.2% ropivacaine for ACB in this study was effective and safe for postoperative analgesia in TKA patients. For continuous adductor canal block, most literature studies had reported the use of ropivacaine at a concentration of 0.2% and an infusion rate of 8 ml/h [34–36]. Veal et al. had described continuous 0.2% ropivacaine infusion at 8 ml/h in a patient who likely had delayed quadriceps weakness within the adductor canal [35]. Neal et al. had presented 3 cases of probable local anesthetic-induced myotoxicity involving CACB with 1.5% lidocaine or 1.5% mepivacaine bolus followed by an infusion of 0.2% ropivacaine [36]. The adductor canal block protected the quadriceps strength by the occurrence of an almost pure sensory nerve block [13, 28]. Zhang et al. had also found that CACB with 0.2% ropivacaine 5 ml/h could effectively be used for analgesia after TKA [37]. Therefore, we performed CACB with 20 ml 0.2% ropivacaine bolus followed by infusion of 0.17% ropivacaine 5 ml/h, which had lower concentration and volume than previous studies [34–36], and had the advantage of high security for postoperative analgesia, and the patients can get out of bed as early as possible.

Surgery and anesthesia could lead to a strong stress response and a significant increase of inflammatory cytokines in patients, which are related to postoperative pain, anxiety, fear, and so on. ESR was a nonspecific inflammatory index, while CRP was a sensitive index for monitoring tissue damage and inflammatory response in clinical practice at present, which was also an important evaluation index in the process of postoperative recovery [38]. IL-6 was a major proinflammatory factor, and its expression level was closely related to the degree of tissue injury caused by surgery [39]. The adjuvant analgesic agents, including celecoxib, parecoxib, and flurbiprofen axetil, which were all some of the nonsteroidal anti‐inflammatory drugs (NSAIDs), were a part of multimodal analgesic treatment for all patients in our study carried out throughout the perioperative period. Klifto et al. had reported that NSAIDs (parecoxib and celecoxib) have been shown to decrease inflammation, pain, and fever [40]. Hu et al. had found that flurbiprofen 100 mg could effectively suppress the elevation of serum interleukin-6 concentration after radical excision of breast cancer [41]. Yang et al. had also reported that adductor canal block combined with cyclooxygenase 2 (COX-2) selective inhibitors (parecoxib and celecoxib) could inhibit the inflammatory response after TKA [42]. As shown in our research, the inflammatory cytokines (ESR, CRP and IL-6) at POH48 in the SACB combined with the PCIA group were lower, which is probably related to the use of celecoxib, parecoxib, and flurbiprofen axetil in PCIA.

In our research, compared with CACB, SACB combined with PCIA provided a larger range of flexion and extension motion of the knee and therefore had achieved better postoperative joint function rehabilitation [15], which remarkably explained the reason for the superiority of the analgesia strategy of SACB combined with PCIA after TKA.

This research also revealed that the analgesia strategy of SACB combined with PCIA had the advantage of the lower postoperative hospital stay and total hospital cost and the higher NRS satisfaction scores at discharge, which was more globally economical than CACB in TKA. All patients in this study have used intravenous dexamethasone 10 mg and tropisetron 2 mg to prevent postoperative nausea and vomiting (PONV). Therefore, the incidence of PONV in SACB combined with the PCIA group (6.4%) was lower and without difference to that in the CACB group (5.1%).

In addition, the total incidence of the complications such as pulmonary infection, cardiovascular events, deep vein thrombosis, incisional infection, and unplanned second surgery in the SACB combined with PCIA group was 1.3%, which was lower than that in the CACB group (5.1%), indicating high safety.

Several limitations to this study should be considered. As a retrospective study, this study has certain biases, a small number of cases, and a short observation time window, which still needs to be confirmed by future studies, such as expanding the sample size, extending the observation time, and carrying out prospective randomized controlled studies.

## 5. Conclusion

In conclusion, ultrasound-guided single-shot adductor canal block combined with patient-controlled intravenous analgesia appeared to provide better analgesia when compared to continuous adductor canal block in the first two days after total knee arthroplasty. It was beneficial for patients in a globally economical manner, inhibited inflammation, and did not increase the incidence of adverse events and complications and thus achieved the purpose of enhanced recovery after surgery.

## Figures and Tables

**Figure 1:** Mean Visual Analogue Scale (VAS) pain scores at rest before operation (Pre) and at postoperative hours (POH), ^#^*P* < 0.05.

**Figure 2:** Mean Visual Analogue Scale (VAS) pain scores with motion before operation (Pre) and at postoperative hours (POH), ^*∗*^*P* < 0.001.

**Figure 3:** Mean range of knee flexion and extension before operation (Pre) and at postoperative hours (POH48), ^*∗*^*P* < 0.001.

**Figure 4:** Mean erythrocyte sedimentation rate (ESR) before operation (Pre) and postoperative 48 hours (POH48), ^#^*P* < 0.05.

**Figure 5:** Mean C-reactive protein (CRP) before operation (Pre) and postoperative 48 hours (POH48), ^#^*P* < 0.05.

**Figure 6:** Mean interleukin-6 (IL-6) before operation (Pre) and postoperative 48 hours (POH48), ^*∗*^*P* < 0.001.

**Table 1:** Demographic and perioperative data.

Characteristic	Group A	Group B	*P* value
Number of patients	78	78	—
Gender (male/female)	17 (22%)/61 (78%)	19 (24%)/59 (76%)	0.850
Age (years)	69.4 ± 7.2	66.9 ± 8.7	0.052
Height (cm)	157.8 ± 6.3	156.9 ± 6.7	0.374
Weight (kg)	62.1 ± 9.9	62.4 ± 8.9	0.806
BMI (kg/m^2^)	24.9 ± 3.6	25.4 ± 3.4	0.401
ASA class (II/III)	26 (33%)/52 (67%)	27 (35%)/51 (65%)	1
Surgery side (left/right)	40 (51%)/38 (49%)	41 (53%)/37 (47%)	1
Length of surgery (min)	77.4 ± 20.5	77.7 ± 15.3	0.923
Length of anesthesia (min)	113.1 ± 28.3	111.6 ± 18.8	0.702
Length of extubation (min)	19.9 ± 9.0	18.8 ± 7.7	0.429
Length of stay in PACU (min)	75.6 ± 14.9	71.5 ± 16.5	0.111
Surgeon (%) (A/B/C/D/E)	15.4/11.5/11.5/35.9/25.6	16.7/6.4/12.8/37.2/26.9	0.865
Anesthetist (A/B)	26 (33%)/52 (67%)	39 (50%)/39 (50%)	0.051

*Note*. Values are presented as mean ± SD or number (percentage). BMI = body mass index; PCIA = patient-controlled intravenous analgesia; ASA = American society of anesthesiologists; PACU = postanesthesia care unit.

**Table 2:** Secondary outcomes.

Characteristic	Group A (*n* = 78)	Group B (*n* = 78)	*P* value
Postoperative first ambulation time (h)	20.8 ± 4.1	20.3 ± 3.9	0.448
Patient-controlled bolus (times)	4.3 ± 1.6	3.1 ± 1.3	≤0.001^*∗*^
Postoperative hospital stay (d)	5.8 ± 1.6	4.7 ± 1.5	≤0.001^*∗*^
Total hospital stay (d)	10.4 ± 2.6	9.6 ± 2.8	0.058
Total hospital cost (RMB)	60496.1 ± 8481.4	56464.9 ± 6045.7	0.001^#^
NRS satisfaction scores at discharge	9.46 ± 0.27	9.66 ± 0.17	≤0.001^*∗*^

*Note*. Values are presented as mean ± SD. PCA = patient-controlled analgesia; NRS = Numerical Rating Scale.^*∗*^*P* < 0.001; ^#^*P* < 0.05.

**Table 3:** Incidence of adverse events and complications.

Characteristic	Group A (*n* = 78)	Group B (*n* = 78)	*P* value
Remedial analgesics treatment (n, %)	9 (11.5%)	5 (6.4%)	0.402
Dizziness, nausea and vomit (n, %)	4 (5.1%)	5 (6.4%)	1
Pulmonary infection (n, %)	2 (2.6%)	0	0.497
Cardiovascular events (n, %)	0	0	1
Deep vein thrombosis (n, %)	2 (2.6%)	1 (1.3%)	1
Incisional infection (n, %)	0	0	1
Unplanned second surgery (n, %)	0	0	1

## Data Availability

The data used and/or analyzed during the current study are available from the corresponding author on reasonable request.
